This article has been retracted.

# Utilizing Entity-Based Gated Convolution and Multilevel Sentence Attention to Improve Distantly Supervised Relation Extraction

**DOI:** 10.1155/2021/6110885

**Published:** 2021-11-01

**Authors:** Qian Yi, Guixuan Zhang, Shuwu Zhang

**Affiliations:** ^1^Beijing Engineering Research Center of Digital Content Technology, Institute of Automation, Chinese Academy of Sciences, Beijing 100010, China; ^2^University of Chinese Academy of Sciences, Beijing 100010, China

## Abstract

Distant supervision is an effective method to automatically collect large-scale datasets for relation extraction (RE). Automatically constructed datasets usually comprise two types of noise: the intrasentence noise and the wrongly labeled noisy sentence. To address issues caused by the above two types of noise and improve distantly supervised relation extraction, this paper proposes a novel distantly supervised relation extraction model, which consists of an entity-based gated convolution sentence encoder and a multilevel sentence selective attention (Matt) module. Specifically, we first apply an entity-based gated convolution operation to force the sentence encoder to extract entity-pair-related features and filter out useless intrasentence noise information. Furthermore, the multilevel attention schema fuses the bag information to obtain a fine-grained bag-specific query vector, which can better identify valid sentences and reduce the influence of wrongly labeled sentences. Experimental results on a large-scale benchmark dataset show that our model can effectively reduce the influence of the above two types of noise and achieves state-of-the-art performance in relation extraction.

## 1. Introduction

The goal of relation extraction is to identify the relationship between two given entities in a sentence. Conventional RE models are trained in a supervised manner with manually labeled data. However, as it is labor intensive to build large-scale manually labeled dataset, the size of the data will limit the effectiveness of the model. So, distant supervision was proposed to solve this problem, in which large-scale labeled data are automatically generated [1].

In distant supervision, a fact triple (*h*, *t*, *r*) of a given knowledge graph (KG) contains the two entities *h* and *t*, where *h, t*, and *r* denote head entity, tail entity, and relation, respectively. Distant supervision will label all sentences containing the two entities *h*and*t* with the relation *r*. Although distant supervision can effectively construct a large-scale relation extraction dataset, it suffers from the inevitable problem of incorrect labeling. This is because not all sentences that contain the entity pair can correctly express the relations in the given KG. For example, given a triple (Bill Gates, Microsoft, and business/company/founders) in a KG and a sentence “Bill Gates retired from Microsoft,” distant supervision will label the sentence with “business/company/founders,” which is clearly an incorrect label.

In addition to the incorrect labeling issue, distant supervision also suffers from the problem of low-quality sentence, which is caused as a result of the dataset being automatically constructed by crawling web pages. We illustrate this issue using the example below. Given the sentence “The problem might have been that the family was in NBC's suite, but Dick Ebersol, the chairman of NBC Universal Sports, said by telephone that…,” we find that the part which expresses the relationship contained in the triple (“Dick Ebersol,” “NBC Universal Sports,” and “/business/person/company”) is the subsentence “but Dick Ebersol, the chairman of NBC Universal Sports.” The other parts of the sentence are meaningless for the relation extraction and may even hinder the performance of the model.

To address these issues, we need to work on the following two fronts: (1) filter out the useless intrasentence noise information when learning sentence representations and (2) reduce the influence of wrongly labeled noisy sentences. For the first aspect, word-level attention has been leveraged to emphasize relational words [2]; however, the effect of useless words cannot be significantly reduced as the proportion of useless words is usually large. Liu et al. [3] proposed the subtree parse (STP) method which intercepts the subtree of each sentence under the lowest common ancestor of the parent entities to remove the useless parts. However, an extraparser is required to preprocess the sentence; hence, the effectiveness of the model will be affected by the performance of the parser. For the second aspect, recent works employed the multi-instance learning (MIL) schema to solve this problem [4, 5]. In these studies, researchers divided sentences into different bag. In each bag, all the sentences contain the same entity pair. And relation extraction proceeds at the bag-level. Furthermore, various extensions of sentence selective attention were proposed to reduce the influence of noise sentences under MIL schema [6–8]. Nevertheless, the semantic information of the whole entity-pair bag is rarely considered in most existing attention-based models. Even for the same relation, different entity pairs express them in different ways. So, the semantic information of the whole entity-pair bag can help to better identify the valid sentences.

In this paper, we propose a novel model for relation extraction to tackle the two types of noise problems introduced by distant supervision. The model is composed of two main modules. One is an entity-based gated convolution sentence encoder. The entity-based gate of the encoder forces the convolution operation to focus on extracting the features related to the entity pair, and the intrasentence noise is filtered out through the pooling operation. After obtaining sentence representations, we apply the second component, the Matt module, to address the problem of wrongly labeled sentences. The Matt module first adopts the original attention mechanism to obtain a first-level bag representation and then fuses it with the query vector through the gated recurrent unit (GRU) to obtain a bag-specific query vector that is aware of the semantic information of the entity-pair bag. Finally, we use the bag-specific query vector to calculate the attention weights and obtain the final bag representation.

The contributions of this paper are summarized as follows:

- To get rid of the influence of the intrasentence noise, we propose an entity-based gated convolution to filter out the useless information and extract entity-pair-related relational features from a sentence
- To address the problem of incorrect labeling, we design a Matt module that generates a bag-specific query vector to assign lower attention scores to those noise sentences
- Experimental results on a large-scale benchmark dataset show that our model can effectively reduce the influence of the above two types of noise and achieve state-of-the-art performance in relation extraction.

The remainder of this paper is organized as follows. In Section 2, we present some related work for open domain relation extraction. In Section 3, we present our proposed relation extraction model. Next, in Section 4, we present experimental results of our model and then analyze the results. Finally, in Section 5, we make a conclusion of our paper and propose our future work.

## 2. Related Work

RE is a fundamental task in natural language processing (NLP). The purpose of relation e-traction is to identify the relationship between two given entities in a sentence. And it can be seen as a kind of text classification task. In text classification, there are two kinds of common methods: the traditional machine learning-based methods [9] and the neural network-based methods [10].

Similarly, RE models can also be divided into above two kinds. Traditional RE methods used manually constructed features and adopted kernel-based classifier to classify the relationship [11, 12]. Recently, neural network-based RE methods have attracted increasing attention. These methods can automatically extract relational features for relation classification and have been found to achieve good performance [2, 13–16]. Some models enhanced the performance of the model by reducing intrasentence noise. Zhou et al. [2] and Jat et al. [17] adopted word-level attention to emphasize relational words and attenuate useless words, but the effect of useless words cannot be significantly reduced for the proportion of useless words that is usually large. Liu et al. [3] built STP to remove noisy words and constructed a neural network inputting the subtree. However, its performance would be affected by the accuracy of the parser.

Like most neural network models, the lack of annotation data limits the performance of these neural relation extraction models. To tackle this problem, distant supervision was proposed to automatically generate large-scale training data for relation extraction [1]. However, this results in the inevitable problem of incorrect labeling. To address this issue, recent works employed MIL schema, in which the relation classification proceeds on bag-level [4, 5, 14, 18]. Moreover, sentence-level attention and its extensions are widely used to reduce the impact of wrong labeled sentences [6, 8, 19]. Apart from these methods, some other selector-based models have also been adapted for RE recently. Reinforcement learning (RL) also was applied to train a binary sentence classifier to remove noise instances [20, 21]. Qin et al. [22] designed a delicate generative adversarial network (GAN), and the classification part is used as a sentence selector. The above methods have alleviated the problem of incorrect labeling to varying degrees.

In this paper, we propose a distantly supervised relation extraction model which is aimed at reducing both intrasentence noise and wrongly labeled noisy sentence. Different from the existing word-level noise reduction models, our model can extract entity-pair-related features and directly filter out the intrasentence noise without the help of any extraparser. As compared with the widely used sentence-level attention model, our Matt module further exploits the bag's semantic information when calculating the attention scores and can better identify valid sentences.

## 3. Method

In this section, we will introduce our distantly supervised relation extraction model in detail. The architecture of our model is shown in Figure 1. The notations and definitions are given as follows.

### 3.1. Notation

Given a KG *G*={*E*, *R*, *F*}, we use *E*, *R*, and *F* to denote entities sets, relations sets, and facts sets. The fact in the knowledge graph refers to the relational triple (*h*,*t*,*r*), indicating that there exists a relation *r* ∈ ℛ between a head entity *h* ∈ *ℰ* and a tail entity *t* ∈ *ℰ*. Following the MIL setting, we divided all sentences into several entity-pair bags {*S*_*h*_1_,*t*_1__,*S*_*h*_2_,*t*_2__,…}. Each bag *S*_*h*_*i*_,*t*_*i*__ contains several sentences {*s*_1_, *s*_2_,…}, in which all the sentences contain the same entity pair (*h*_*i*_,*t*_*i*_). The distant supervision labels the entity-pair bag *S*_*h*_*i*_,*t*_*i*__ with the corresponding relation *r*_*i*_ in the fact triple (*h*_*i*_,*r*_*i*_,*t*_*i*_). Each sentence *s* is composed of a sequence of words *s*={*w*_1_,*w*_2_,…}.

### 3.2. Overall Framework

Given an entity pair (*h*_*i*_,*t*_*i*_) and its corresponding entity-pair bag *S*_*h*_*i*_,*t*_*i*__, the relation extractor aims to obtain the probability *P*(*r|h*_*i*_,*t*_*i*_,*S*_*h*_*i*_,*t*_*i*__) of each relation *r* ∈ ℛ existing between *h*_*i*_ and *t*_*i*_.

As shown in Figure 1, our relation extractor is composed of two modules: an entity-based gated convolution sentence encoder and a Matt module. First, the entity-based gated convolution sentence encoder encodes each sentence *s*_*i*_ in the entity-pair bag *S*_*h*_*i*_,*t*_*i*__ into a low-dimensional, fixed-length vector **s**_*i*_. Then, to reduce the impact of wrongly labeled sentences in each bag, we adopt a Matt module to assign an attention weight *α*_*i*_ for each sentence *s*_*i*_. After obtaining the sentence representations and their corresponding attention weights, we calculate the weighted sum of sentence representations as the bag representation **r**_*h*_*i*_,*t*_*i*__ for the entity-pair bag:

(1) $$\begin{array}{c} r_{h_{i},t_{i}}=\sum \alpha_{j}s_{j}. \end{array}$$

Finally, we feed the bag representation to the linear projection and softmax function to obtain the conditional probability *P*(*r|h*_*i*_,*t*_*i*_,*S*_*h*_*i*_,*t*_*i*__) for each relation *r*:

(2) $$\begin{array}{c} o=W\cdot r_{h_{i},t_{i}},\\ P\left(r|h_{i},t_{i},S_{h_{i},t_{i}}\right)=\frac{\exp\;o_{r}}{\sum_{k=1}^{n_{r}}\exp\;o_{k}}, \end{array}$$

where *W* is the weight matrix and *n*_*r*_ is the relation number.

### 3.3. Entity-Based Gated Convolution Sentence Encoder

Given a sentence *s*={*w*_1_,*w*_2_,…} and the entity pair (*h*,*t*), we employ the entity-based gated convolution sentence encoder to extract relational features for relation classification.

#### 3.3.1. Input Layer

Firstly, we feed the given sentence *s* into the input layer to embed *s* into a matrix, which contains both semantic and positional information of each word.

*(1) Word Embedding*. Word embeddings are low-dimensional, continuous, and real-valued vectors, which can capture semantic meanings of words. They can embed each word in the vocabulary into a vector **v**_*w*_ ∈ *R*^*d*_*w*_^. In this paper, we use the New York Times (NYT) corpus to train the word embedding with the Skip-Gram [23] algorithm.

*(2) Position Embedding*. Position embeddings can capture the positional information of each word. We utilize the relative position between each token and the two target entities to indicate the position of the token. For example, in the sentence “Yao Ming was born in Shanghai,” the relative position from the word born to the target entity Yao Ming is 2 and to Shanghai −2. Position embeddings embed each relative position value into a vector **v**_*p*_ ∈ *R*^*d*_*p*_^.

We concatenate the word embedding *v*_*w*_ and two position embeddings (each corresponds to one target entity) **v**_*p*_en 1__ and **v**_*p*_en 2__ to get the word representation **v** ∈ *R*^*d*_*w*_+*d*_*p*_*∗*2^. Given a sentence *s*={*w*_1_,…, *w*_*n*_} with *n* words, we concatenate all words representations to obtain an embedding matrix C={*v*_1_; …; *v*_*n*_}.

#### 3.3.2. Entity-Based Gated Convolution

The entity-based gated convolution is composed of a gated convolution layer and a pooling layer.

*(1) Gated Convolution Layer*. The gated convolution layer consists of two convolution units. One of them is a plain convolution unit; the other is an entity-based convolution operation. In the plain convolution, a convolution kernel **W**_*s*_ ∈ ℛ^*d*_*v*_×*m*×*k*^ slides through the embedding matrix **C**, where *d*_*v*_=*d*_*w*_+*d*_*p*_*∗*2 is the dimension of the word representation, *m* is the size of convolution kernel, and *k* is the dimension of the output. The *k*-dimensional hidden features are calculated as follows:

(3) his=Re LUvi−m−1/2,…,vi+m−1/2⊗Ws+bs,

where ⊗ denotes the convolution operation.

Regarding the entity-based convolution, an entity-related component *W*_en_ · *v*_en_^*T*^ is added to the original convolution operation. **W**_en_ ∈ *R*^*k*×2*∗d*_*v*_^ is a weight matrix, and **v**_en_=*w*_en_1__*w*_en_2__ ∈ *R*^2*∗d*_*v*_^ is the concatenation of the embedding vectors of two entities *w*_en_1__ and *w*_en_2__. The entity-related hidden features are calculated as follows:

(4) $$\begin{array}{c} h_{i}^{\text{en}}=\sigma \left(\left[v_{i-\left(m-1\right)/2},...,v_{i+\left(m-1\right)/2}\right]⊗W_{g}+W_{\text{en}}\cdot v_{\text{en}}+b_{g}\right), \end{array}$$

where *σ* represents the sigmod function, **W**_*g*_ ∈ *R*^*d*_*v*_×*m*×*k*^ is the convolution kernel, and *b*_*g*_ ∈ *R*^*k*^ is a bias. Then, the entity-based gated convolution feature vector is obtained by computing an element-wise multiplication between **h**^*s*^ and **h**^en^:

(5) $$\begin{array}{c} h_{i}^{g}=h_{i}^{s}⊙h_{i}^{\text{en}}, \end{array}$$

where ⊙ denotes element-wise multiplication. Through the operation in equation (5), the entity-related features **h**^en^ function as a controlling gate to force the gated convolution operation to extract relational features that relate to a given entity pair. Then, an entity-based gated convolution feature map **H**^*g*^={**h**_1_^*g*^; **h**_2_^*g*^; …} is fed to the pooling layer.

*(2) Pooling Layer*. For the pooling layer, two alternatives are adopted: the traditional max-pooling and the piecewise max-pooling. In the following sections, we will abbreviate entity-based gated convolution with max-pooling and piecewise max-pooling as entity-based gated convolution network (EGCNN) and entity-based gated piecewise convolution network (EGPCNN), respectively. The traditional max-pooling operation selects the maximum value of each row of the feature map *H*^*g*^ to obtain the final feature vector:

(6) $$\begin{array}{c} q_{j}=\underset{1\leq j\leq n}{\max}\left\{h_{i,j}\right\}. \end{array}$$

Piecewise max-pooling is a variant of the traditional max-pooling operation:

(7) $$\begin{array}{c} q_{j}^{\left(1\right)}=\underset{1\leq j＜i_{\text{en }1}}{\max}\left\{h_{i,j}\right\},\\ q_{j}^{\left(2\right)}=\underset{i_{\text{en }1}\leq j＜i_{\text{en }2}}{\max}\left\{h_{i,j}\right\},\\ q_{j}^{\left(3\right)}=\underset{i_{\text{en }2}＜j\leq n}{\max}\left\{h_{i,j}\right\}, \end{array}$$

in which the subscript *j* denotes the *j*-th element of a vector and *i*_en 1_ and *i*_en 2_ are the positions of two entities. Then, three pooling vectors are concatenated to get the final sentence representation as follows:

(8) $$\begin{array}{c} q_{j}=\left\{q_{j}^{\left(1\right)},q_{j}^{\left(2\right)},q_{j}^{\left(3\right)}\right\}. \end{array}$$

### 3.4. Multilevel Sentence Selective Attention

After encoding sentences with the sentence encoder, we obtain the sentence representations {**s**_1_, **s**_2_,…} for each entity-pair bag *S*_*h*,*t*_={*s*_1_,*s*_2_,…}. We adopt a multilevel sentence selective attention to generate attention weight for each sentence.

We first obtain the first-level bag embedding via the original sentence-level attention mechanism. The attention weight *β* for each sentence is calculated as follows:

(9) $$\begin{array}{c} e_{i}=q_{r}^{T}W_{a}s_{i},\\ \beta_{i}=\frac{\exp\left(e_{i}\right)}{\sum_{j}^{N}\exp\left(e_{j}\right)}, \end{array}$$

where **W**_*a*_ ∈ *R*^*d*_*v*_×*d*_*v*_^ is the weight matrix, *N* is the number of sentences, and **q**_*r*_ is the query vector assigned for the relation *r*. Accordingly, we obtain the bag embedding **r** by calculating the weighted sum of sentence representations as in equation (1). To simplify the notion, we abbreviate the operations for calculating the attention weight in equation (9) as follows:

(10) $$\begin{array}{c} \text{ATT}\left(q_{r},s\right), \end{array}$$

where the first element **q**_*r*_ denotes the query vector and the second element **s** denotes the sentence representations.

After obtaining the first-level bag embedding, we adopt a nonlinear operation to fuse the semantic information in the bag embedding **r** into the original query vector **q**_*r*_ to obtain a bag-specific query vector.

In particular, we employ GRU to update the original query vector. Given the original query vector **q**_*r*_ and the first-level bag embedding **r**, the bag-specific query vector **q**_*r*_^*b*^ is calculated as follows:

(11) $$\begin{array}{c} r=\sigma \left(W_{r}r+U_{r}q_{r}\right), \end{array}$$

(12) $$\begin{array}{c} z=\sigma \left(W_{z}r+U_{z}q_{r}\right), \end{array}$$

(13) $$\begin{array}{c} {\tilde{q}}_{r}^{b}=\tan\;h\left(W_{x}r+W_{g}\left(r⊙q_{r}\right)\right), \end{array}$$

(14) $$\begin{array}{c} q_{r}^{b}=\left(1-z\right)⊙q_{r}+z⊙{\tilde{q}}_{r}^{b}, \end{array}$$

where **W**_*r*_, **W**_*z*_, **U**_*r*_, **U**_*z*_, and **W**_*x*_ ∈ ℛ^*d*_*v*_×*d*_*v*_^. As we can see from equations (13) and (14), the state of the bag-specific query vector *q*_*r*_^*b*^ is the interpolation of the original query vector **q**_*r*_ and the bag embedding **r**. Thus, the bag-specific query vector contains both the relational information and the whole bag's semantic information, which can be adopted to provide more fine-grained sentence selection.

Then, we calculate the bag-specific attention score *α*_*i*_ for sentence *s*_*i*_ as follows:

(15) $$\begin{array}{c} \alpha_{i}=\text{ATT}\left(q_{r}^{b},s_{i}\right). \end{array}$$

Accordingly, with the bag-specific attention scores {*α*_1_,*α*_2_,…} and the sentence representations {**s**_1_, **s**_2_,…}, we can compute the final bag embedding **r**_*h*,*t*_ using equation (1). The bag embedding **r**_*h*,*t*_ is fed to the linear projection, and the softmax function is used to calculate the conditional probability *P*(*r|h*,*t*,*S*_*h*,*t*_) following equation (2).

### 3.5. Training

We employ the negative log likelihood as loss for our model. Given a collection of sentence bags Ω={*S*_*h*_1_,*t*_1__,*S*_*h*_2_,*t*_2__,…} and corresponding labeling relation {*r*_*i*_,*r*_2_,…}, the loss is defined as follows:

(16) $$\begin{array}{c} ℒ=-\frac{1}{\left|\Omega \right|}\sum_{i=1}^{\left|\Omega \right|}\log\;p\left(r_{i}|h_{i},t_{i},S_{h_{i},t_{i}},\theta \right), \end{array}$$

where |Ω| is the number of bags. To optimize our model, we apply Adam optimizer [24] to minimize the loss in equation (16).

## 4. Result and Discussion

### 4.1. Dataset and Evaluation

Following the existing literature, we evaluate our model on the New York Times (NYT) dataset developed by Riedel et al. [4]. The NYT dataset is constructed by aligning Freebase with NYT corpus through distant supervision. The training set and the test set contain 522611 and 172448 sentences, separately. These sentences are divided into 53 candidate categories. There is a label “NA” in these 53 relations, indicating that there is no relationship between two target entities. During training, we randomly select 10% of the sentences from the training data as the validation data.

We evaluate all methods via the held-out evaluation, which compares the relational facts extracted from the test set by the models with all the facts existing in the test set. For evaluation, we present precision-recall curves for all models. Furthermore, we also report the Precision@N results of all models .

### 4.2. Implementation Detail

1. In the experiment, we set most of the experimental parameters according to Lin et al. [6]. We also utilize dropout on the fully connected layers in our model to avoid overfitting. The detailed experimental parameter value settings used in our experiments are summarized in Table 1. For model training, we adopt Adam optimizer to update the model. We conduct experiments on two NVIDIA GTX K40. The algorithm is written in python in Ubuntu 16.04 system.

### 4.3. Comparison with Previous Models

In order to evaluate the effectiveness of our relation extraction model, we compare it with five recent representative models:

 
*PCNN* *+* *MIL.* This work [18] proposed piecewise convolution network (PCNN) to obtain sentence representations and utilized the MIL framework to solve the noise problem
 
*PCNN* *+* *ATT*. This work [6] used piecewise convolution network to obtain sentence vectors and adopted the attention mechanism to alleviate the impact of noise sentence
 
*STP.* This work [3] built a subtree parse method to reduce intrasentence noise and constructed a neural network inputting the subtree while applying entity-wise attention to identify the important semantic features
 
*PCNN* *+* *PU*. This work [25] applied RL to construct positive and unlabeled bag and improve the distantly supervised relation extraction model with positive and unlabeled (PU) learning.
 
*JOINT_PCNN* *+* *RL*. This work [26] introduced a RL framework to jointly train a sentence-level relation extraction model

We evaluate all the competing models and our proposed models (EGPCNN + Matt and EGPCNN + ATT) via held-out evaluation and report their performances with the precision-recall curve in Figure 2.

From the results, we can observe the following :

1. When compared with the two baseline models: PCNN + MIL and PCNN + ATT, our models exhibit a significant improvement. It indicates that the two well-designed components in our model can assist in extracting a more delicate bag representation and improve the performance of relation extraction. Furthermore, we will discuss the effects of each component in Section 4.4.
2. Our EGPCNN + ATT model steadily outperforms STP, which takes measures to reduce the influence of the intrasentence noise, in precision-recall curve. This result indicates that, as compared with models which removes noise words with extraparser, our entity-based gated convolution operation can improve the extraction of effective features and directly filter out intrasentence noise.
3. EGPCNN + Matt also outperforms the PCNN + PU and JOINT_PCNN + RL model. PCNN + PU is a novel work that adopts RL and makes full use of positive and unlabeled bags. JOINT_PCNN + RL also utilizes reinforced learning but to train the sentence encoder. This demonstrates the effectiveness of our model, which can eliminate the noise in both word and sentence level.
4. Table 2 shows P@N for relation extraction using variable number of sentences in bags (with more than one sentence). Here, one, two, and all represent the number of sentences randomly selected from a bag. We can observe that the EGPCNN + Matt model achieves the best result among all models. Especially in the experiment of all sentence situation, the EGPCNN + Matt model shows apparent advantage, which indicates our model can better filter out noise information when there are large amounts of instances and retain more useful information.

### 4.4. Effect of Various Model Components

In this section, we conduct more experiments to further evaluate the effects of different components in our model.

#### 4.4.1. Effect of the Entity-Based Gated Convolution

To evaluate the effect of the entity-based gated convolution, we compare the performances of the following three models: (1) PCNN with sentence-level attention (PCNN + ATT), (2) gated PCNN with sentence-level attention (GPCNN + ATT), and (3) entity-based gated PCNN with sentence-level attention (EGPCNN + ATT). The difference between the second and the third models is that the second model removes the entity-related component *W*_en_ · *v*_en_^*T*^ from equation (4).

We display the performances of above models with precision-recall curves in Figure 3. From Figure 3, we can obtain the following: (1) EGPCNN + ATT significantly outperforms the other two models, which indicates that the entity-based gated convolution operation is effective at extracting entity-pair-related features and can help improve the relation extraction performance; (2) GPCNN + ATT, which removes the entity-related component, has no improvement when compared with the PCNN + ATT. It demonstrates that the entity-related component *W*_en_ · *v*_en_^*T*^ is a crucial part to the gated convolution operation. Without the entity information in the entity-related component, the convolution gate cannot filter out the intrasentence noisy information.

To further verify that the entity-based gated convolution can extract better sentence representations, we conduct experiments on the sentence-level relation classification task. We randomly chose 300 sentences and manually labeled the relation type for each sentence to construct a test set. We consider each sentence as an entity-pair bag with only one sentence; the attention weight for the sentence is 1, and the bag representation is identical to the sentence representation. We adopt CNN + ATT and PCNN + ATT as baseline models and compare their performances with EGCNN + ATT and EGPCNN + ATT, both of which add an entity-based gated convolution component on the basis of the two baseline models. We adopted accuracy and macroaveraged F1 as the evaluation metric.

As shown in Table 3, EGCNN + ATT and EGPCNN + ATT outperform CNN + ATT and PCNN + ATT by 0.16 and 0.07 in macroaveraged F1 and 0.06 and 0.07 in accuracy, respectively. These results further verify that the entity-based gated convolution operation can eliminate the influence of useless words and extract sentence representations better than the convolution operation without entity-based gate.

#### 4.4.2. Effect of the Multilevel Sentence Selective Attention

To evaluate the effect of the multilevel sentence selective attention in our model, we adopt PCNN + ATT and EGPCNN + ATT as baseline. We combine the two baseline models with the Matt module and utilize the PR curve to evaluate the performances of four models: PCNN + ATT, EGPCNN + ATT, PCNN + Matt, and EGPCNN + Matt.

Figure 4 shows that PCNN + Matt and PECNN + Matt outperform PCNN + ATT and PECNN + ATT separately. This result demonstrates that multilevel sentence selective attention can eliminate the effects of noisy sentences more effectively than the original attention, and the multilevel attention mechanism will not be influenced by the structure of the sentence encoder.

Figure 5 shows the effect of different layer number for the PCNN + Matt model. From the results, we can find out that the two-layer structure achieves the best performance. When the layer number continues to increase, the performance of model declines.

## 5. Conclusion and Future Work

In this paper, we propose a novel distantly supervised relation extraction model. It can effectively address the problems of the intrasentence noise and the wrongly labeled sentence. The entire model contains an entity-based gated convolution sentence encoder and a Matt module. The entity-based gated convolution operation forces the sentence encoder to pay more attention to the entity-pair-related parts of the sentence and filters out the useless information. The multilevel sentence selective attention considers information of the whole bag when generating the attention weights and helps in producing improved bag representation. We conduct the experiments on a widely used dataset. Experimental results verify the effectiveness of the two modules, and our model achieves state-of-the-art results.

Except the methods used in the paper, some of the most representative computational intelligence algorithms can also be used to solve the problem, like Slime mould algorithm (SMA) [27] and Harris hawks optimization (НHO) [28]. Different from these models, our model proposes the Matt to reduce the sentence-level noise and the EGPCNN to reduce the inner-sentence noise and improve the performance of RE.

In the future, we plan to adopt extra information like entity description and sentence syntax information to help extract more precise entity-pair-related relational features. Furthermore, we will combine our attention model with recent selector-based denoising methods to address the problem of wrongly labeled sentence. These selector-based denoising methods train a sentence classifier to further remove the wrongly labeled sentence and can further improve our model.

## Figures and Tables

**Figure 1:** Architecture of our model. The overall structure of our model is in the left, the details of sentence encoder and Matt are in the middle, and details of the entity-based gated convolution operation are on the right.

**Figure 2:** Comparison with representative models.

**Figure 3:** Comparison between PCNN + ATT, GPCNN + ATT, and EGPCNN + ATT.

**Figure 4:** Comparison between PCNN + ATT, EGPCNN + ATT, PCNN + Matt, and EGPCNN + Matt.

**Figure 5:** Performance comparison between different number of attention layers.

**Table 1:** Experimental parameter settings.

Batch size	Learning rate	Maximum sentence length	Hidden layer dimension for CNNs	Word dimension	Position dimension	Convolution kernel size	Dropout rate
50	0.001	120	230	50	5	3	0.5

**Table 2:** P@N for relation extraction using variable number of sentences in bags (with more than one sentence).

P@N	One				Two				All			
	100	200	300	Mean	100	200	300	Mean	100	200	300	Mean
PCNN + MIL	0.73	0.65	0.57	0.650	0.70	0.67	0.63	0.667	0.72	0.70	0.64	0.687
PCNN + ATT	0.73	0.69	0.61	0.677	0.77	0.72	0.66	0.717	0.76	0.73	0.67	0.720
STP	0.83	0.76	0.67	0.752	0.85	0.81	0.72	0.794	0.87	0.83	0.78	0.827
PCNN + PU	0.87	0.76	0.70	0.777	0.89	0.79	0.72	0.799	0.90	0.82	0.77	0.828
JOINT_RL	0.86	0.75	0.71	0.773	0.87	0.80	0.74	0.803	0.88	0.83	0.76	0.830
EGPCNN + ATT	0.85	0.78	0.69	0.773	0.86	0.81	0.73	0.800	0.89	0.83	0.78	0.833
EGPCNN + Matt	0.88	0.78	0.73	0.797	0.88	0.83	0.75	0.820	0.90	0.85	0.80	0.850

**Table 3:** Performance comparison of different sentence encoders on the sentence-level relation extraction task.

Method	Macro F1	Accuracy
CNN + ATT	0.30	0.58
EGCNN + ATT	0.46	0.64
PCNN + ATT	0.45	0.66
EGPCNN + ATT	0.52	0.73

## Data Availability

The data used to support this study are available in the website: https://catalog.ldc.upenn.edu/LDC2008T19.
